The article "Information System Security Evaluation Algorithm Based on PSO-BP Neural Network" was retracted in 2023. Reasons: suspected computer-generated content; unreliable results or conclusions; concerns about the data; concerns about the results or conclusions.

# Information System Security Evaluation Algorithm Based on PSO-BP Neural Network

**DOI:** 10.1155/2021/6046757

**Published:** 2021-08-17

**Authors:** Qinghua Zheng

**Affiliations:** School of Business, Jinling Institute of Technology, Nanjing 211169, Jiangsu, China

## Abstract

With the deepening of big data and the development of information technology, the country, enterprises, organizations, and even individuals are more and more dependent on the information system. In recent years, all kinds of network attacks emerge in an endless stream, and the losses are immeasurable. Therefore, the protection of information system security is a problem that needs to be paid attention to in the new situation. The existing BP neural network algorithm is improved as the core algorithm of the security intelligent evaluation of the rating information system. The input nodes are optimized. In the risk factor identification stage, most redundant information is filtered out and the core factors are extracted. In the risk establishment stage, the particle swarm optimization algorithm is used to optimize the initial network parameters of BP neural network algorithm to overcome the dependence of the network on the initial threshold, At the same time, the performance of the improved algorithm is verified by simulation experiments. The experimental results show that compared with the traditional BP algorithm, PSO-BP algorithm has faster convergence speed and higher accuracy in risk value prediction. The error value of PSO-BP evaluation method is almost zero, and there is no error fluctuation in 100 sample tests. The maximum error value is only 0.34 and the average error value is 0.21, which proves that PSO-BP algorithm has excellent performance.

## 1. Introduction

Information system is widely used in finance, construction, information security, and other fields. With the increasing amount of information and the rising price of information, there is no lack of criminals stealing valuable information [1]. However, information security risk assessment started later than that in Europe and America, especially in the late 20th century. With the continuous improvement of science and technology, more and more information security issues threaten the information environment security. In this case, more and more scholars began to study related technologies. Oliveira et al. proposed a multichannel decision-tree-based method for power system operation security assessment. Different from other decision tree techniques, in the training step, a value of classification attribute is established according to branches, which improves the interpretability of power system operation state because operators can clearly see the key variables of each topology, so they can use MDT rules to assist decision-making. The results show that the MDT method simplifies the power system security classification and has good accuracy [2]. Sun et al. proposed a new feature extraction framework based on deep learning, which is used to build the risk assessment model. The depth automatic encoder is used to convert the space of conventional state variables into a small number of dimensions, so as to optimally distinguish safe operation from unsafe operation. Through a series of case studies and comparisons, the superior performance of the framework is proved, and it is mapped to IEEE 118 bus system [3].

Benini and Sicari [4] took the lead in focusing on security risk assessment in cloud computing and released relevant research reports in 2008, summarizing the seven security risks affecting cloud computing services. Then Mantri et al. [5] analyzed the risks of Haas, PAAS, and SaaS in the cloud computing architecture from other perspectives. In 2014, based on the existing scientific research, Jiang and Yang [6] summarized the risk factors affecting the security of cloud computing services. In addition, scholars from various countries have also carried out in-depth research. Chiang et al. [7] have studied the information risk elements faced by networks and information systems and proposed an object-oriented management information base model to configure the access rights of each file to improve security risks by evaluating the risks encountered by autonomous communication networks. Patil et al. [8] used the fault tree model in engineering to conduct in-depth analysis and security risk assessment of information systems and strives to objectively and truly express the security performance of information systems. Wiesche et al. [9] combined with his many years of theoretical research and practical experience, theoretically discussed the principle and future development trend of information security risk assessment. With the development of Internet technology, various threats have sounded an alarm to people. From the painful lessons, people understand that we should comprehensively protect the information system, avoid all possible risks and reduce the possibility of information security events. In recent years, some scholars began to apply parallel PSO-BP neural network algorithm. Hou et al. [10] proposed parallel PSO-BP neural network algorithm. PSO algorithm is used to optimize the initial weights and thresholds of BP neural network to improve the accuracy of classification results. The results show that compared with the traditional serial PSO-BP neural network algorithm, the classification accuracy of parallel PSO-BP neural network algorithm is about 92%, and the system efficiency is about 0.85, which has obvious time and classification effect when processing large data sets. Gu et al. [11] applied particle swarm optimization BP neural network prediction model to SiCp/Al composite grinding energy consumption prediction model. The results show that particle swarm optimization (PSO) BP neural network prediction model has high prediction accuracy. The energy consumption prediction model based on PSO-BP neural network is conducive to energy saving and green manufacturing. Lin et al. [12] established a sensor error correction model based on particle swarm optimization (PSO) and BP neural network algorithm, which reduced the nonlinear characteristics of the system and improved the test accuracy of the system. Simulation and experiments show that PSO-BP neural network algorithm has the advantages of fast convergence speed and high diagnosis accuracy and can provide higher measurement accuracy, lower power consumption, stable network data communication, and fault diagnosis functions. It has been applied to the monitoring of environmental parameters, such as warehouses, special vehicles, and ships. Moayedi et al. [13] proposed the PSO-BP risk assessment system, which transfers the object instance called by the user to the storage device on the hardware layer of the network information system, and the object is carried by the tenant of the network information service. Information system is widely distributed in all walks of life, and its position is becoming more and more important. In the past research, few studies can organically combine intelligent learning algorithm with information system risk assessment to monitor information system risk in real time. Therefore, this paper will improve the intelligent learning BP algorithm, combined with PSO algorithm, to realize the intelligent risk assessment of information system and establish the information system protection framework.

Using the advantages of simple principle, fast convergence speed and less parameter setting of PSO algorithm, the initial weight threshold of principal component neural network is optimized, and the algorithm flow of principal component neural network based on particle swarm optimization is established. The algorithm is applied to information security risk assessment, and compared with the information security risk assessment algorithm based on BP neural network. MATLAB simulation results show that the improved algorithm has higher prediction accuracy than the traditional BP neural network algorithm.

## 2. Information Security Risk Assessment Based on BP Neural Network Optimized by PSO Algorithm

### 2.1. Improved BP Neural Network Prediction Model

In the evaluation of information system security, there are many data and strong correlation between them. Due to the lack of analysis and processing ability of input data, the classical BP neural network algorithm is relatively complicated in training structure, which is not conducive to the fitting of the network. Therefore, it needs to be slightly improved [14–17]. In this paper, principal component analysis method is used to remove the correlation between risk factors, reduce the dimension of multiple risk data indicators, linearly transform multiple variables of risk factors indicators, retain most of the original information, and finally get the core component which can represent the original data information, and then input it into BP neural network as the initial data, Avoid the influence of repeated information in the evaluation [18–20]. Correspondingly, due to the reduction of input data, the input nodes of BP neural network are also reduced correspondingly, the system is simplified, the data relationship is relatively simple and the same, the convergence speed of the system is faster, and it also has a positive impact on the prediction accuracy. The improved BP neural network is shown in Figure 1.

Suppose there are *n* samples in the two-dimensional space, and the distribution of samples is shown in Figure 2(a). It can be seen that in the plane where these samples are located, the discrete type is very large no matter which direction they are in. If the analysis is carried out only from the *X* or *Y* direction, the necessary information will be lost in the coordinate axis, which will have a great impact on the evaluation results [21, 22]. After transformation, Figure 2(b) is obtained from Figure 2(a), and the transformation formula is shown in the following formula:

(1) $$\begin{array}{c} \left\{\begin{array}{c} X^{\prime }=X\;\cos\;\theta +Y\;\sin\;\theta ,\\ -Y^{\prime }=-X\;\cos\;\theta +Y\;\sin\;\theta , \end{array}\right. \end{array}$$

After transformation, new variables *X*′ and *Y*′ are obtained. It is not difficult to see that the dispersion degree of *Y*′ sample in the coordinate system *X*′ − *Y*′ is obviously lower than *X* − *Y*, while the dispersion degree of *X*′ sample is higher than *Y*′ sample, which can almost represent all the information of important data. The data are relatively complete. That is to say, the influence of data characteristics in *X*′ direction on the evaluation results is very small and can be ignored. The matrix expression is shown as follows:

(2) $$\begin{array}{c} \left[\begin{array}{c} X^{\prime }\\ Y^{\prime } \end{array}\right]=\left(\begin{array}{c} \begin{array}{cc} \cos\;\theta & \sin\;\theta \end{array}\\ \begin{array}{cc} -\sin\;\theta & \cos\;\theta \end{array} \end{array}\right)\left[\begin{array}{c} X\\ Y \end{array}\right]=U\left[\begin{array}{c} X\\ Y \end{array}\right]. \end{array}$$

In information system security evaluation, the *i*th target quantity is composed of *N* factors. Then, the *n*-dimensional vector *X*=(*X*_1_, *X*_2_, ..., *X*_*n*_), linear change *x*, gets *y*, and *Y*=(*Y*_1_, *Y*_2_, *Y*_3_, ..., *Y*_*m*_), which is the comprehensive variable of security information. The expression is shown as follows:

(3) $$\begin{array}{c} \left\{\begin{array}{c} Y_{1}=\alpha_{11}X_{1}+\alpha_{12}X_{2}+\cdots +\alpha_{1n}X_{n}\\ Y_{2}=\alpha_{21}X_{1}+\alpha_{22}X_{2}+\cdots +\alpha_{2n}X_{n}\\ Y_{3}=\alpha_{m1}X_{1}+\alpha_{m2}X_{2}+\cdots +\alpha_{mn}X_{n} \end{array}\right\}, \end{array}$$

where *X* is the factor, *α* is the coefficient, the coefficients *α*_*ij*_ satisfy *α*_*i*1_^2^+*α*_*i*2_^2^+⋯*α*_in_^2^=1,  *i*=1,2,…, *n*, and *Y*_*i*_ satisfy *D*(*Y*_1_) > *D*(*Y*_2_) > …>*D*(*Y*_*m*_). In addition, there is no linear relationship between *Y*_*i*_ and *Y*_*j*_, *i* ≠ *j*. Considering the above variable conditions, we can obtain a change matrix A of order *n* × *n*, as follows:

(4) $$\begin{array}{c} A=\left[\begin{array}{cccc} \alpha_{11} & \alpha_{12} & \ldots & \alpha_{1n}\\ \alpha_{21} & \alpha_{22} & \ldots & \alpha_{2n}\\ \ldots & \ldots & \ldots & \ldots \\ \alpha_{n1} & \alpha_{n2} & \ldots & \alpha_{nn} \end{array}\right]. \end{array}$$

After the linear change of the initial variable *X*_1_, *X*_2_,…, *X*_*n*_, a new principal component variable *Y*_1_, *Y*_2_,…, *Y*_*n*_ is obtained, which is not related to each other. The expression between the two can be expressed as follows:

(5) $$\begin{array}{c} Y=\left[Y_{1},Y_{2},\ldots ,Y_{n}\right]=A^{T}X. \end{array}$$

The determination of the number of principal components *m* value is mainly realized through the gravel map and the cumulative contribution of principal components. In the case of the determination of principal components, the greater the cumulative contribution rate of the first *m* principal components indicates that these principal components contain most of the effective information, and the smaller the probability of information loss. The standard *X*_*i*×*j*_ is obtained by the normalization of the following formula:

(6) $$\begin{array}{c} \left\{\begin{array}{c} x_{ij}^{'}=\frac{x_{ij}-M_{j}}{S_{j}},\\ M_{j}=\frac{1}{n}\sum_{i=1}^{n}x_{ij},\\ S_{j}=\sqrt{\frac{1}{n-1}\sum_{i=1}^{n}{\left(x_{ij}-M_{j}\right)}^{2}}, \end{array}\right. \end{array}$$

where *S*_*j*_ represents the two-level fuzzy comprehensive evaluation matrix and *M*_*j*_ represents the model function. The covariance matrix *D* is obtained from the standardized data, as shown in the following formula:

(7) $$\begin{array}{c} D=\frac{1}{n-1}X^{T}X, \end{array}$$

where *n* is the number of samples and the eigenvalue matrix *L* and eigenvector matrix A of *D* are calculated by formula (7), with RA = RL. Finally, the matching principal component is selected to replace the initial data and input to BP neural network. The calculation of matrix A is to solve the contribution rate and cumulative contribution rate of the *k*th principal component according to the eigenvalue *λ*, and the calculation formula is shown as follows:

(8) $$\begin{array}{c} \left\{\begin{array}{c} \text{ratio}=\frac{\lambda_{k}}{\sum_{j=1}^{n}\lambda_{j}},\\ \text{sum}=\sum_{j=1}^{k}\frac{\lambda_{k}}{\sum_{j=1}^{n}\lambda_{j}}. \end{array}\right. \end{array}$$

Among them, ratio and sum represent contribution rate and cumulative contribution rate, respectively.

### 2.2. Particle Swarm Optimization Algorithm Based on Principal Element Neural Network

In this study, the particle swarm optimization algorithm is used to optimize the initial parameters of the principal component neural network, overcome the shortcomings of the network, such as strong dependence on the initial value, slow learning rate and falling into local minimum, and establish an information security risk assessment model based on particle swarm optimization principal component neural network. Although the BP neural network algorithm optimized by input nodes has been simplified to a certain extent, it is not different from the traditional BP algorithm in global optimization ability. Both of them are easy to fall into local minimum and affect global optimization. Generally speaking, as long as the weights and thresholds of the neural network can be optimized, the problem of local minimum can be avoided [23, 24]. Part of the research combines genetic algorithm with BP neural network using the powerful macro search ability and good global optimization performance of genetic algorithm. However, the operation of genetic algorithm is complex, which needs a series of processes such as selection, replication, crossover, and mutation, which greatly reduces the training speed of neural network. The PSO algorithm has higher convergence performance than the genetic algorithm, combined with BP algorithm can inherit its high prediction accuracy, and further accelerate the convergence speed of the improved BP algorithm [25]. The particle in PSO algorithm is the weight and threshold that need to be optimized in BP algorithm, and the particle dimension *D* is the number of them. Generally speaking, the smaller the *w* is, the faster the convergence speed of the algorithm is. But at the same time, it is also necessary to avoid the PSO particles falling into the local optimal state in the optimization and iteration. The larger the *w* is, the easier it is to fall into the local optimal state. Therefore, considering the two factors, the change of *w* value is set to decrease gradually. Initialize the attributes of *N* particles, as shown in the following formulae:

(9) $$\begin{array}{c} \begin{array}{cc} v_{j}=\left[v_{j1},v_{j2},\ldots ,v_{j\;D}\right] & x_{j}=\left[x_{j1},x_{j2},\ldots ,x_{j\;D}\right] \end{array}, \end{array}$$

(10) $$\begin{array}{c} p_{j}=\begin{array}{cc} \left[p_{j1},p_{j2},\ldots ,p_{j\;D}\right] & p_{g}=\left[p_{g1},p_{g2},\ldots ,p_{g\;D}\right] \end{array}. \end{array}$$

Among them, *v*_*i*_, *x*_*i*_, *p*_*i*_, and *p*_g_ represent the velocity, position, optimal position, and optimal position of particle swarm, respectively. The inertia weight method is used to update the velocity of particles, and the calculation formula is shown in following formula:

(11) $$\begin{array}{c} w\left(t\right)=w_{\max}-\frac{w_{\max}-w_{\min}}{T_{\max}}t=0.9-\frac{t}{2T_{\min}}, \end{array}$$

Among them, *c*, *r*, *v*(*t*), and *x*(*t*) represent the learning factor, random number of [0,1] interval, particle velocity, and particle position respectively; *w*(*t*), *t*, and *T*_max_ represent inertia weight, number of iterations, and maximum number of iterations respectively, and the value of learning factor is 2 [26, 27]. The update of velocity is constrained by the limited value of particle velocity and calculated according to the following formulae:

(12) $$\begin{array}{c} r\left(x\right)=\left\{\begin{array}{cc} v_{\max} & x>v_{\max}\\ -v_{\max} & x<-v_{\max}\\ x & \left|x\right|\leq v_{\max} \end{array}\right., \end{array}$$

(13) $$\begin{array}{c} x\left(t+1\right)=r\left(v\left(t+1\right)\right). \end{array}$$

At this time, the particle position is updated, that is, there is *x*(*t*+1)=*x*(*t*)+*v*(*t*+1). Finally, the optimal position of each particle and the optimal position of the population are updated through the fitness function *f*(*∗*). The update formulae are shown as follows:

(14) $$\begin{array}{c} p_{i}\left(t+1\right)=\left\{\begin{array}{cc} p_{i}\left(t\right), & f\left(p_{i}\left(t\right)\right)\leq f\left(x_{i}\left(t+1\right)\right),\\ x_{i}\left(t+1\right), & f\left(p_{i}\left(t\right)\right)>f\left(x_{i}\left(t+1\right)\right), \end{array}\right. \end{array}$$

(15) $$\begin{array}{c} \begin{array}{cc} p_{g}\left(t+1\right)=p_{i}\left(t+1\right) & f\left(p_{i}\left(t+1\right)\right) \end{array}=\min f\left(p\left(t+1\right)\right). \end{array}$$

If the maximum number of iterations is met, the result will be output. Otherwise, it is necessary to jump to the inertial update particle velocity step again until the conditions are met. The detailed flowchart is shown in Figure 3.

To sum up, the overall idea of PSO algorithm to optimize BP algorithm is to first clarify the topological layer structure of BP neural network, continuously screen out the optimal weights and thresholds through PSO algorithm, and then give BP neural network, finally train the samples to be learned and the corresponding expectations, and finally get the prediction results of test samples.

### 2.3. Establishment of BP Neural Network Security Evaluation Model Optimized by PSO

As the core content of organizations, enterprises, and institutions, the value of information is immeasurable, and a little error may bring irreparable losses, so we need to implement comprehensive protection for it fundamentally. The premise of information security risk assessment of information system is to classify its most media assets scientifically and reasonably, which is the cornerstone of risk assessment.  Figure 4 shows the detailed classification of information assets of information system.

The security of information assets consists of the security of information confidentiality, integrity, and availability. To ensure the security of the three elements, the security characteristics of asset information can be mapped in the information security risk assessment. However, in the era of big data, the storage mode and value of information are completely different from those in the past. With the popularity of the network, information may have security vulnerabilities and be illegally invaded. Therefore, in the information security risk assessment, it is necessary to consider the different requirements of the three elements of the assets in the business process from the perspective of information assets and levels. According to the impact on the information system when the security of three elements is attacked, three different threat levels are given to the different threat elements of three elements of information assets. The detailed classification is shown in Figure 5.

In Figure 5, Level A represents a high threat, that is, it is very important. The destruction of this security attribute often brings great losses to the owner; Level B indicates medium threat, that is, relatively important. If this security attribute is damaged, it may cause moderate loss; C means low threat. The damage of this security attribute will bring less loss to the owner. It can be seen that among the confidentiality attributes, the most important one is the important secrets of the organization/enterprise; in integrity, the most important is the information with the highest integrity value. The most important attribute of usability is the information that the organization/enterprise often uses every day, accounting for 90% or more, and the interruption time is required to be less than 10 minutes. If the above information is modified or destroyed without authorization, it may cause serious losses to the organization/enterprise. The fragility is used to evaluate the security of information system, that is, the difficulty of the system being attacked by the outside world and causing damage to the system under normal operation. The mainstream international common vulnerability assessment system (CVSS) is used to grade the system. Class A is highly brittle, indicating that there is a big loophole or it is easy to be broken, so it needs to be rectified and reinforced immediately; Class B is of medium fragility, which needs to be attached great importance and repaired or reinforced when necessary; Class C is low brittleness, which needs to be paid attention to and reinforced or repaired when appropriate.

As an example of the hierarchical structure model of the evaluated information system shown in Figure 6, the risk factors of the information system are listed one by one, and the occurrence of information security accidents is regarded as the top event of the fault tree. There are three situations: the threat of the information system, the weakness of the information system itself, and the existing security measures. The fault tree corresponding to the hierarchical structure model is established. Due to the high confidentiality of information security risk assessment and the nonlinear fuzzy state among the risk assessment factors, it is difficult to obtain the typical sample data, especially the risk factors such as assets, threats, and vulnerability. To verify the scientificity and effectiveness of the model in information security risk assessment, 80 evaluation samples of CNCERT are selected as the simulation experimental data. After selecting data samples, the algorithm modeling of PSO-optimized PCA neural network is carried out, and the specific steps are shown in Figure 6.

## 3. Simulation Results Analysis of Information Security Risk Assessment Based on PSO-Optimized PCA Neural Network

### 3.1. Performance Analysis of PSO-BP Neural Network Algorithm

Algorithm performance analysis is performed in Windows 10(86×) platform. The software used for this analysis is Python. To compare the convergence performance, running speed and accuracy of BP neural network algorithm, PSO algorithm, genetic algorithm, GA-PSO, and PSO-BP algorithm under the premise of the same error target, the error is set to 10 to 5, and the maximum number of cycles is set to 20000. There are 45,800 sets of experimental data, of which 10000 are data that need to be identified and evaluated, including asset identification, fragility identification, threat identification, and identification of existing security measures. The convergence performance of the five algorithms is shown in Figure 7.

As can be seen from Figure 7, the convergence of the four algorithms is quite different. Among the three different training samples, the convergence of BP algorithm is the worst, the number of iterations exceeds 4000, and it falls into local optimum in two more complex training, with an average running time of 365.9 seconds. The convergence of PSO algorithm is close to that of GA algorithm. In the three experiments, both of them converge about 2000 times. However, compared with the running time, the running time of GA algorithm is significantly higher than that of PSO algorithm, which is 683 seconds for the former and 124.3 seconds for the latter. The reason is that GA algorithm has more operation processes and needs multiple selection, crossover, and mutation operations, which is more complex than PSO algorithm. Therefore, it takes a long time to run. PSO-BP neural algorithm is excellent in terms of convergence speed and running speed. The four sample training iterations are completed in about 500 times, and the average running time is only 183.6 seconds. For GA-BP algorithm, although the convergence of the optimization algorithm is very similar to PSO-BP algorithm, but in terms of running time, the combination of the two can reach 1078.0 seconds, which seriously affects the efficiency of the system. In the PSO-BP algorithm, BP algorithm inherits the accuracy and fast optimization ability of PSO algorithm, so it has better advantages than GA-BP algorithm in overall performance, which also shows that it is reasonable for PSO algorithm to optimize BP neural network algorithm. It can be seen that PSO-BP neural algorithm is superior to other algorithms in terms of time and efficiency and has high cost-effectiveness.

### 3.2. Analysis of Simulation Results of Information Security Risk Assessment

Eighty risk factor sets are selected as the evaluation samples, and a single sample contains 14 risk factors, that is to determine the risk factor matrix R80 × 14, and then preprocess the elements in the matrix to reduce the potential unreasonable influence. After removing the correlation between risk factors, the lithotripsy diagram and principal component contribution diagram are shown in Figure 8(a).

It can be seen that five of the 14 eigenvalues are greater than or equal to 1. From the curve change trend, the curve curvature of the principal component fraction from 1 to 9 is significantly greater than that of 9 to 14. Combined with the analysis of contribution (Figure 8(b)), when the number of principal components extracted is greater than or equal to 7, the cumulative contribution rate has exceeded 90%, covering most of the information of the initial 14 factors. It shows that the influence of the other seven factors on the system evaluation results can be ignored, and the original 14 data can be replaced by seven principal components. The risk assessment results of the algorithm before and after optimization are shown in Figure 9.

In 88 samples, it can be seen that the error rate of the unoptimized BP algorithm is obviously high, and it is easy to misjudge, especially for the judgment of Class A risks. Specifically, the BP neural algorithm misjudges 8 Class A risks in the firewall serious loopholes, communication system faults and special faults as Class C risks; The denial of service attack, file loss and other 8 Class B risk events are misjudged as normal events; five Class C risks such as operation error and weak password are misjudged as a risk; eight normal events were misjudged as risk events. However, the algorithm optimized by PSO has only one misjudgment, that is, a Level A risk event is determined as a Level C risk event, which has high accuracy on the whole. Through literature search, it is concluded that the currently more effective and commonly used objective evaluation methods are PSO algorithm and BP neural network. The comparison of the objective evaluation results and subjective evaluation scores of the two networks and PSO-BP is shown in Figure 8. The detailed error bars are shown in Figure 10.

It can be seen from Figure 10 that the highest score of experts for 100 information system security is 9.8, and the lowest is 6.9. The deviaion between BP neural network scoring and expert scoring is serious. The coincidence degree of the scoring results of PSO algorithm and the subjective evaluation results of experts is much higher than that of BP neural network scoring. The score curve of the improved PSO-BP evaluation method is almost the same as that of the experts, which shows that the score of the improved PSO-BP evaluation method is closer to the subjective evaluation of the experts. The two neural networks are compared with PSO-BP in objective evaluation and subjective evaluation error values, and the comparison results are shown in Figure 11.

From the error curve, the PSO neural network has less fluctuation, better fit with the actual value, and has more advantages in the whole network structure, and the learning and training process of PSO algorithm is simpler than that of BP neural network. Therefore, in the objective evaluation, although the BP neural network evaluation error for most of the samples is small, the maximum error value of BP neural network is 3.87, the error value between the sample number 41∼71 fluctuates the most, the average error value during the period is as high as 2.76, and the total average error value is 1.48. The maximum error value of PSO algorithm is 1.12, and there is no area with large error fluctuation, and its average error value is 0.84, so on the whole, the error value of PSO algorithm is smaller and more stable, and its performance is better. It is not difficult to see that the error value of PSO-BP evaluation method is almost zero, and there is no error fluctuation in 100 sample tests. The maximum error value is only 0.34, and the average error value is 0.21, which is far less than the average error value of 1.48 of BP neural network evaluation and 0.84 of PSO algorithm evaluation. The stability of PSO-BP evaluation method in evaluating the security of information system is obviously better than other network evaluation methods, and its error range is very small and can be almost ignored.

## 4. Conclusion

Information security risk assessment is very important to ensure the normal operation of information system, and the selection of scientific and reasonable risk assessment method is the primary task of efficient and scientific information security risk assessment. As for the current risk assessment method, on the basis of qualitative analysis, quantitative synthesis is used again, and the organic combination of the two has been widely used.

The rapid development of information technology, increasingly convenient information system and developed and flexible information network have gradually become an important pillar supporting human society in the information age, and the accompanying problem is information security. More and more people understand the importance and urgency of information security. As an important part of information security management, information security risk assessment has also attracted the attention of relevant institutions and researchers. Choosing an efficient and reasonable risk assessment method is very important for information security risk assessment, especially for the smooth progress of the assessment work. Taking advantage of the advantages of PSO, such as simple principle, fast convergence speed, and less parameter setting, the initial weight threshold of principal component neural network is optimized, and the algorithm flow of principal component neural network based on particle swarm optimization is established. The algorithm is applied to information security risk assessment and compared with the information security risk assessment algorithm based on BP neural network. The simulation results of MATLAB show that the improved algorithm has higher prediction accuracy than the traditional BP neural network algorithm. There are too many risk factors involved in the process of information security risk assessment. In addition, a formal risk assessment needs to spend a huge amount of money, and the data of risk assessment is highly confidential, which leads to a certain complexity and difficulty of this scientific research. Only through hard exploration, accumulation, and careful improvement can we find information security risk assessment and prediction algorithms with high precision, wide range, and strong adaptability, and provide basis for better information system security management decision-making and security strategy formulation.

Using the advantages of simple principle and fast convergence speed of PSO, this paper optimizes the traditional BP neural network, reduces its dependence on initial threshold and weight, speeds up the learning speed and reduces the probability of falling into local extremum, and establishes the PSO-BP algorithm. Compared with the traditional BP algorithm, the algorithm proposed in this paper converges faster, runs faster, and has better accuracy. In the simulation experiment, the error of PSO-BP algorithm in predicting the risk of information system is almost 0, the error of traditional BP algorithm is 3.87, and the maximum error of PSO algorithm is 1.12. It shows that PSO-BP algorithm can accurately evaluate the security of information system. In the process of information system security risk assessment, there are many risk factors, huge investment amount, and the assessed data are highly confidential, which makes the research in this field more difficult. Only by continuously improving the technology and exploring the assessment methods with stronger adaptability, wider scope, and better accuracy, can we better provide security management decisions for information system security.

Due to time constraints, this paper only uses fewer data samples. If more data samples, such as historical risk assessment data, can be collected, a small information security risk assessment database can be constructed. When conducting risk assessment for a certain type of information system, the risk assessment data samples that meet the characteristics of this kind of information system can be extracted to train and verify the assessment algorithm model, so as to increase the fairness, accuracy, and reliability of the assessment results.

## Figures and Tables

**Figure 1:** Improved BP neural network algorithm at input.

**Figure 2:** Discrete form of particles. (a) Distribution of sample in *X*-*Y*. (b) Distribution of sample in *X*′-*Y*′.

**Figure 3:** Flowchart of BP neural network optimized by PSO.

**Figure 4:** Asset information classification.

**Figure 5:** Three elements assignment of information assets.

**Figure 6:** Information system security risk assessment model.

**Figure 7:** Convergence performance of five algorithms. (a) First training. (b) Second training. (c) Third training. (d) Algorithm.

**Figure 8:** (a) Principal component analysis. (b) Principal component contribution rate.

**Figure 9:** Sample validation. (a) Unoptimized BP neural network and (b) BP neural network optimized by PSO.

**Figure 10:** Comparison of different neural network expert scoring.

**Figure 11:** Error comparison of three neural networks.

## Data Availability

The data used to support the findings of this study are available from the corresponding author upon request.
